The article "Mechanisms of quadriceps muscle weakness in knee joint osteoarthritis: the effects of prolonged vibration on torque and muscle activation in osteoarthritic and healthy control subjects" was published in 2011. Journal: Arthritis Res Ther.

# Mechanisms of quadriceps muscle weakness in knee joint osteoarthritis: the effects of prolonged vibration on torque and muscle activation in osteoarthritic and healthy control subjects

**DOI:** 10.1186/ar3467

**Published:** 2011-09-20

**Authors:** David A Rice, Peter J McNair, Gwyn N Lewis

**Affiliations:** 1 Health and Rehabilitation Research Institute, AUT University, 90 Akoranga Drive, Northcote, 0627 Auckland, New Zealand

## Abstract

**Introduction:**

A consequence of knee joint osteoarthritis (OA) is an inability to fully activate the quadriceps muscles, a problem termed arthrogenic muscle inhibition (AMI). AMI leads to marked quadriceps weakness that impairs physical function and may hasten disease progression. The purpose of the present study was to determine whether γ-loop dysfunction contributes to AMI in people with knee joint OA.

**Methods:**

Fifteen subjects with knee joint OA and 15 controls with no history of knee joint pathology participated in this study. Quadriceps and hamstrings peak isometric torque (Nm) and electromyography (EMG) amplitude were collected before and after 20 minutes of 50 Hz vibration applied to the infrapatellar tendon. Between-group differences in pre-vibration torque were analysed using a one-way analysis of covariance, with age, gender and body mass (kg) as the covariates. If the γ-loop is intact, vibration should decrease torque and EMG levels in the target muscle; if dysfunctional, then torque and EMG levels should not change following vibration. One-sample *t *tests were thus undertaken to analyse whether percentage changes in torque and EMG differed from zero after vibration in each group. In addition, analyses of covariance were utilised to analyse between-group differences in the percentage changes in torque and EMG following vibration.

**Results:**

Pre-vibration quadriceps torque was significantly lower in the OA group compared with the control group (*P *= 0.005). Following tendon vibration, quadriceps torque (*P *< 0.001) and EMG amplitude (*P *≤0.001) decreased significantly in the control group but did not change in the OA group (all *P *> 0.299). Hamstrings torque and EMG amplitude were unchanged in both groups (all *P *> 0.204). The vibration-induced changes in quadriceps torque and EMG were significantly different between the OA and control groups (all *P *< 0.011). No between-group differences were observed for the change in hamstrings torque or EMG (all *P *> 0.554).

**Conclusions:**

γ-loop dysfunction may contribute to AMI in individuals with knee joint OA, partially explaining the marked quadriceps weakness and atrophy that is often observed in this population.

## Introduction

Individuals with osteoarthritis (OA) of the knee joint commonly display marked weakness of the quadriceps muscles, with strength deficits of 20 to 45% compared with age and gender-matched controls [1-3]. Persistent quadriceps weakness is clinically important in individuals with OA as it is associated with impaired dynamic knee stability [4] and physical function [2,3,5]. Moreover, the quadriceps have an important protective function at the knee joint, working eccentrically during the early stance phase of gait to cushion the knee joint and acting to decelerate the limb prior to heel strike, thereby reducing impulsive loading [6,7]. Weaker quadriceps have been associated with an increased rate of loading at the knee joint [7,8], and recent longitudinal data have shown that greater baseline quadriceps strength may protect against incident knee pain [9,10], patellofemoral cartilage loss [9] and tibiofemoral joint space narrowing [11].

The article "Mechanisms of quadriceps muscle weakness in knee joint osteoarthritis: the effects of prolonged vibration on torque and muscle activation in osteoarthritic and healthy control subjects" was published in 2011. Journal: Arthritis Res Ther.

There are many causes of quadriceps weakness in OA patients, some of which are not fully understood. However, an important determinant of this weakness is arthrogenic muscle inhibition (AMI) - an ongoing neural inhibition that prevents the quadriceps muscles from being fully activated [12-14]. As well as being a direct cause of quadriceps weakness [13], AMI may contribute to muscle atrophy [15] and, in more severe cases, can prevent effective quadriceps strengthening [16-18]. There are several lines of evidence to suggest that AMI is caused by a change in the discharge of sensory receptors from the damaged knee joint [14,15,19]. In turn, a change in afferent discharge may alter the excitability of multiple spinal reflex and supraspinal pathways that combine to limit activation of the quadriceps α-motoneuron pool (for a review see [14]). A strong increase in knee joint mechanoreceptor and/or nociceptor discharge (as with acute swelling, pain or inflammation) leads to marked quadriceps AMI [20-22]. However, some patients with knee joint pathology continue to display striking quadriceps activation deficits in the absence of pain and clinically detectable effusion [19,23,24]. Furthermore, there is evidence from animal studies that different populations of knee joint mechanoreceptors have opposing effects on quadriceps α-motoneuron pool excitability and that in the normal, uninjured knee the net effect may be excitatory [25-27]. Thus, it is possible that a loss of normal sensory output from a population of excitatory knee joint mechanoreceptors also contributes to AMI.

One of the neural pathways thought to be involved in mediating AMI is the γ-loop (Figure 1). The γ-loop is a spinal reflex circuit formed by γ-motoneurons innervating muscle spindles that in turn transmit excitatory impulses to the homonymous α-motoneuron pool via Ia afferent nerve fibres.

The article "Mechanisms of quadriceps muscle weakness in knee joint osteoarthritis: the effects of prolonged vibration on torque and muscle activation in osteoarthritic and healthy control subjects" was published in 2011. Journal: Arthritis Res Ther.

**Figure 1:** **Schematic diagram of the γ-loop**. During voluntary muscle contraction, supraspinal centres coactivate the α-motoneuron and γ-motoneuron pools. The γ-motoneuron pool in turn innervates muscle spindle endings via fusimotor nerve fibres, enhancing their firing. Muscle spindles provide a tonic excitatory input to the homonymous α-motoneuron pool via Ia sensory nerve fibres.

Hagbarth and colleagues were the first to demonstrate that excitatory input from Ia afferents is necessary to achieve full muscle activation [28]. These authors showed that preferential anaesthetic block of γ-efferents reduced the firing rate of tibialis anterior motor units during subsequent maximum-effort voluntary contractions (MVCs). These changes could be partially reversed by experimentally enhancing spindle discharge from the affected muscle. Further investigations into the importance of the γ-loop have relied on prolonged vibration to experimentally attenuate the afferent portion of the γ-loop. A vibratory stimulus, applied to the muscle or its tendon, temporarily dampens transmission in Ia afferent fibres by increasing presynaptic inhibition, raising the activation threshold of Ia fibres and/or causing neurotransmitter depletion at the Ia afferent terminal ending [29].

In healthy subjects, prolonged vibration (20 to 30 minutes) causes a reduction in muscle force output [30-33], electromyography (EMG) activity [30,32,33] and motor unit firing rates [30] during subsequent MVCs. In people who have ruptured their anterior cruciate ligament (ACL), however, prolonged vibration has no effect on quadriceps muscle activation [32]. Similar observations have since been confirmed up to 20 months after ACL reconstruction [34-36]. These findings suggest that ACL rupture causes an impairment in normal Ia afferent feedback (termed γ-loop dysfunction) that limits quadriceps α-motoneuron depolarisation [32]. It is thought that γ-loop dysfunction is caused by a loss of sensory output from damaged mechanoreceptors within the injured knee joint [32]. Given the notable tissue degeneration present in osteoarthritic knees, a loss of sensory output from a portion of knee joint mechanoreceptors seems likely. The purpose of the current study was therefore to determine whether quadriceps γ-loop dysfunction is also present in individuals with knee joint OA.

## Materials and methods

### Subjects

Fifteen subjects with OA of the knee joint (Kellgren Lawrence Score ≥2) and 15 control subjects with no history of knee injury or pathology volunteered to participate in this laboratory-based study. Subjects from both groups responded to an advertisement requesting volunteers for research examining muscle weakness in people with knee joint OA. All volunteers in the patient group had ongoing knee pain and had previously been diagnosed with OA by their general practitioner. We did not attempt to match OA subjects to control subjects on a case by case basis. However, the control subjects were selected so that the two groups were similar in terms of age and gender (see Table 1). Volunteers in both groups were excluded if they had a previous history of lower limb or spinal surgery, back pain in the past 6 months with associated neurological signs or symptoms, or any pathology that precluded their participation in maximum-effort strength testing. Subjects provided written informed consent for all experimental procedures. Ethical approval for the present study was granted by the Auckland University of Technology Ethics Committee (Auckland, New Zealand) in accordance with the principles set out in the declaration of Helsinki.

The article "Mechanisms of quadriceps muscle weakness in knee joint osteoarthritis: the effects of prolonged vibration on torque and muscle activation in osteoarthritic and healthy control subjects" was published in 2011. Journal: Arthritis Res Ther.

**Table 1:** Participant characteristics

Characteristic	Osteoarthritis group	Control group
Age (years)	63.0 (9.7)	62.4 (10.5)
Height (m)	1.69 (0.10)	1.70 (0.07)
Mass (kg)	77.4 (16.9)	70.0 (9.1)
Female	8 (53.3%)	8 (53.3%)
Dominant limb tested	9 (60.0%)	9 (60.0%)
Radiographic knee osteoarthritis^a^		
Grade II	4 (26.7%)	-
Grade III	6 (40.0%)	-
Grade IV	5 (33.3%)	-
Medial compartment	13 (86.7%)	-
Lateral compartment	9 (60.0%)	-
Patellofemoral compartment	11 (73.3%)	-
Bilateral knee osteoarthritis	6 (40.0%)	-

Data presented as mean (standard deviation) or *n *(%). No significant between-group differences were found for age, height or mass (all *P *≥0.186). ^a^More symptomatic knee in patients with bilateral osteoarthritis.

### Radiographic assessment

Subjects in the OA group were required to have a radiograph of the affected knee joint within 2 weeks of testing. Weight-bearing, fixed flexion radiographs of the knee were taken in the posteroanterior and lateral views [37] and were scored by a single radiologist according to the Kellgren Lawrence scale [38]. Only subjects with a Kellgren Lawrence Score ≥2 were included in the study.

### Experimental setup

All subjects performed a standardised, 5-minute warm-up on an exercycle. Thereafter, subjects were seated in a custom-designed chair with the hips and knees flexed to 90°. Straps were firmly secured over the distal third of the thigh and across the chest to limit extraneous movement. A rigid strap was secured around the ankle, slightly superior to the malleoli. This was coupled to a metal attachment that was connected in series to a uniaxial load cell (Precision Transducers, Auckland, New Zealand), aligned horizontally with the ankle joint.

The article "Mechanisms of quadriceps muscle weakness in knee joint osteoarthritis: the effects of prolonged vibration on torque and muscle activation in osteoarthritic and healthy control subjects" was published in 2011. Journal: Arthritis Res Ther.

### Quadriceps and hamstrings maximum voluntary isometric contractions

Strength testing procedures were undertaken in the (most) affected limb of the OA subjects and the matched limb (dominant/nondominant) of the healthy controls. All subjects were asked to perform MVCs of their quadriceps and hamstrings muscles by pushing or pulling as hard as possible against the ankle strap. Prior to maximum-effort contractions, a series of four submaximal quadriceps and four submaximal hamstrings contractions (25%, 50%, 50% and 75% of perceived maximum effort) were performed, with a 1-minute rest given between each contraction. Thereafter, a 2-minute rest was given before a set of three (6-second) quadriceps MVCs were performed followed by three (6-second) hamstrings MVCs. Subjects received a consistent level of verbal encouragement [39] and were given a 2-minute rest period between each maximum-effort contraction. In the event that the peak force (N) produced during MVCs continued to increase with each subsequent trial, a fourth and in some cases a fifth contraction was performed until force plateaued or decreased. This was done in an effort to elicit a true maximum effort from each individual. Force (N) signals were recorded from the load cell during each contraction, where they were amplified (x100), sampled (1,000 Hz) and displayed in real time on a computer monitor placed in front of the subject using a customised software programme (Testpoint 7; Measurement Computing Corporation, Norton, MA, USA)

### Surface electromyography

During each MVC, surface EMG signals were collected from the vastus medialis, vastus lateralis, semitendinosus and biceps femoris muscles. Prior to the placement of electrodes, the skin was shaved, abraded and cleaned with alcohol to reduce signal impedance. Bipolar AgCl electrodes (Norotrode 20; Myotronics Inc., Kent, WA, USA) were positioned over the target muscles in accordance with the Surface Electromyography for the Non-Invasive Assessment of Muscles guidelines [40]. A ground electrode (Red Dot; 3 M, St Paul, MN, USA) was positioned over the proximal tibia. All EMG signals were amplified (x1,000), filtered (10 to 1,000 Hz) (AMT-8; Bortec Biomedical, Calgary, Alberta, Canada), and sampled at 2,000 Hz (Micro 1401; Cambridge Electronic Design, Cambridge, UK).

### Vibration protocol

Following the initial set of quadriceps and hamstrings MVCs, subjects were asked to relax and remained seated in the chair with their hips and knees flexed to 90°. Vibration was then applied to the infrapatellar tendon using an electrodynamic shaker (Ling Dynamic Systems, Royston, UK), controlled by a customised software program (Signal 3; Cambridge Electronic Design, Cambridge, UK) (Figure 2). Vibration was maintained for 20 minutes at a frequency, amplitude and force of 50 Hz, 1.5 mm and 25 to 30 N, respectively [32,36]. Subjects were asked to remain as still as possible during the application of vibration. The leg was clamped in place for the duration of the vibration period to prevent movement of the tendon relative to the vibration probe. Immediately after vibration, subjects performed another set of at least three quadriceps MVCs and three hamstrings MVCs, in an identical manner to that described above. To avoid potential bias, subjects were kept unaware of the hypothesis of the study and the purposes of the vibration until after their final post-vibration MVC. Hamstrings MVCs were included in the present study to provide evidence that our vibration protocol was specific to the quadriceps muscles and that the vibration did not affect the activation of other muscles in the surrounding area.

The article "Mechanisms of quadriceps muscle weakness in knee joint osteoarthritis: the effects of prolonged vibration on torque and muscle activation in osteoarthritic and healthy control subjects" was published in 2011. Journal: Arthritis Res Ther.

**Figure 2:** **Experimental setup used during vibration of the infrapatellar tendon**.

### Data analysis

At each measurement interval, peak isometric quadriceps and hamstrings strengths were calculated as the highest force (N) produced during any of the three to five MVCs performed for each muscle group. The length of the lever arm was measured from the lateral epicondyle of the femur to the centre of the ankle strap, which was parallel to the load cell. The lever arm length (m) was then multiplied by the peak isometric force (N) to calculate the peak torque (Nm).

Using specialised software (Signal 3; Cambridge Electronic Design, Cambridge, UK), the root mean square (RMS) of the EMG signals from each muscle were calculated from a 1-second period corresponding to the time of maximum activation for each contraction.

### Statistical analysis

Shapiro-Wilk tests were completed to assess whether the dependent variables conformed to a normal distribution (and thus whether parametric testing could be undertaken). Student's *t *tests were used to analyse differences in baseline characteristics between the OA and control groups. Between-group differences in pre-vibration quadriceps and hamstrings peak torque (Nm) were analysed using an analysis of covariance, with body mass (kg), age and gender as the covariates [41]. If the γ-loop is intact, vibration should decrease torque and EMG levels in the target muscle, usually by 7 to 15% [29,32]. If dysfunctional, then torque and EMG levels should not change following vibration. One-sample *t *tests were thus undertaken to analyse whether percentage changes in quadriceps and hamstrings torque and RMS differed from zero after vibration in each group. In addition, analyses of covariance were undertaken to analyse between group differences in the percentage change in quadriceps and hamstrings torque and RMS following vibration. The covariates were age, gender and mass. The significance level for all statistical procedures was set to 0.05.

The article "Mechanisms of quadriceps muscle weakness in knee joint osteoarthritis: the effects of prolonged vibration on torque and muscle activation in osteoarthritic and healthy control subjects" was published in 2011. Journal: Arthritis Res Ther.

## Results

### Baseline characteristics

Baseline characteristics for each group are presented in Table 1. There was no statistically significant difference in age (*P *= 0.686), height (*P *= 0.844) or mass (*P *= 0.186) between groups (Table 1). Results of the Shapiro-Wilk tests suggested that each of the dependent variables was normally distributed (all *P *> 0.08). Pre-vibration quadriceps peak torque was significantly lower in the OA group (mean = 121 Nm; 95% confidence interval = 95, 147 Nm) compared with the control group (mean = 177 Nm; 95% confidence interval = 151, 203 Nm) (*P *= 0.005). While hamstrings peak torque was lower in the OA group compared with the control group, this difference did not reach statistical significance (*P *= 0.101) (Figure 3).

**Figure 3:** **Pre-vibration quadriceps and hamstrings peak torque (Nm) in the osteoarthritis and control groups**. MVC, maximum voluntary isometric contraction at 90° of knee flexion. *Significant difference between groups (*P *= 0.005). Data are means and standard deviations.

### Changes in peak torque following tendon vibration

A summary of peak torque values at each measurement interval is presented in Table 2. Following tendon vibration, a statistically significant decrease in quadriceps peak torque was observed in the control group (*P *< 0.001) but not in OA subjects (*P *= 0.299) (Figure 4). The change in quadriceps torque was significantly different between groups (*P *= 0.011). After vibration, the change in hamstrings peak torque did not differ from zero in either the OA group (*P *= 0.586) or the control group (*P *= 0.902) and the change in hamstrings torque was not different between groups (*P *= 0.670).

**Table 2:** Summary of dependent variables pre and post vibration in each group

Dependent variable	Group	Pre vibration	Post vibration	Change (%)
Quadriceps PT*	OA	128 ± 49	124 ± 44	-2.4
	Control	170 ± 59	156 ± 55	-8.2**
Vastus medialis RMS*	OA	0.13 ± 0.06	0.13 ± 0.06	1.4
	Control	0.27 ± 0.19	0.24 ± 0.18	-13.3**
Vastus lateralis RMS*	OA	0.13 ± 0.06	0.13 ± 0.06	3.9
	Control	0.22 ± 0.13	0.19 ± 0.13	-14.1**
Hamstrings PT	OA	48 ± 18	49 ± 16	1.7
	Control	56 ± 19	55 ± 19	-0.4
Semitendinosus RMS	OA	0.17 ± 0.09	0.18 ± 0.10	7.1
	Control	0.22 ± 0.12	0.23 ± 0.15	3.8
Biceps femoris RMS	OA	0.12 ± 0.10	0.10 ± 0.08	-2.5
	Control	0.16 ± 0.07	0.16 ± 0.07	2.6

Data presented as mean ± standard deviation. OA, osteoarthritis; PT, peak torque (Nm); RMS, root mean square of electromyographic signals. *Significant difference between groups (*P *< 0.05). **Significant change from zero (*P *< 0.05).

The article "Mechanisms of quadriceps muscle weakness in knee joint osteoarthritis: the effects of prolonged vibration on torque and muscle activation in osteoarthritic and healthy control subjects" was published in 2011. Journal: Arthritis Res Ther.

**Figure 4:** **Change in quadriceps and hamstrings peak torque following vibration**. Percentage change in quadriceps and hamstrings peak torque (Nm) following vibration in the osteoarthritis and control groups. *Significant difference between groups (*P *= 0.011). **Significant change from zero (*P *< 0.05). Data are means and standard error of the means.

### Changes in surface electromyography following tendon vibration

A summary of RMS values at each measurement interval is presented in Table 2. After vibration, a statistically significant decrease in vastus medialis RMS was observed in the control group (*P *< 0.001) but not in OA subjects (*P *= 0.786) (Figure 5). Similarly, vastus lateralis RMS decreased after vibration in the control group (*P *= 0.001), but not in the OA group (*P *= 0.466). Significant between-group differences were observed for changes in vastus medialis RMS (*P *= 0.005) and vastus lateralis RMS (*P *= 0.001). After vibration, the change in semitendinosus and biceps femoris RMS values did not differ from zero in either the OA group or the control group (all *P *≥0.204) and the changes did not differ between groups (both *P *≥0.554).

**Figure 5:** **Change in quadriceps surface electromyography amplitude following vibration**. Percentage change in quadriceps surface electromyography (EMG) amplitude following vibration in the osteoarthritis and control groups. RMS, root mean square of EMG signals; VL, vastus lateralis; VM, vastus medialis. *Significant difference between groups (*P *≤0.005). **Significant change from zero (*P *≤0.001). Data are means and standard errors of the means.

## Discussion

The findings of the present study suggest that γ-loop dysfunction contributes to quadriceps AMI in individuals with knee joint OA. Prolonged tendon vibration induces a temporary γ-loop dysfunction by impairing the afferent transmission from Ia fibres to the homonymous α-motoneuron pool [29]. The subsequent loss of excitatory sensory input reduces α-motoneuron excitability, preventing full activation of the muscle. A decrease in quadriceps peak torque and RMS values is thus expected after vibration, as observed in the control group. In contrast, the lack of change in quadriceps activation seen in the OA group suggests that Ia afferent transmission may have already been impaired in these individuals, thus torque and EMG amplitude were unaffected by vibration. This is in accordance with previous findings from populations who had ruptured their ACL [32] or recently had an ACL reconstruction [36,42].

γ-loop dysfunction probably occurs due to a change in sensory output from the damaged knee joint. Studies in animals have established that stimulation of knee joint afferents can elicit strong reflex effects on γ-motoneurons of the muscles surrounding the knee [43-45]. Furthermore, the facilitation of extensor γ-motoneurons is blocked when knee joint afferents are anaesthetised [43]. These observations have led to suggestions that structural damage to the knee joint may simultaneously damage the sensory receptors located in these tissues, disrupting their normal afferent output. In turn, this may diminish quadriceps γ-motoneuron excitability and impair Ia afferent firing, preventing full activation of the muscle [19,46]. In support of this conjecture, Konishi and colleagues observed a reduction in maximum quadriceps torque production and EMG amplitude following the injection of 5 ml local anaesthetic into uninjured human knee joints [32]. In patients who had ruptured their ACL, however, anaesthetising the knee joint had no effect on quadriceps torque and EMG [47]. Furthermore, these authors showed that prolonged vibration failed to reduce quadriceps muscle activation in subjects with uninjured but anaesthetised knee joints.

γ-loop dysfunction may thus occur due to structural changes in the OA joint such as soft tissue degeneration of the ligaments and joint capsule [48,49] or altered capsular compliance [20,50] that reduce excitatory output from mechanoreceptors in the knee joint to quadriceps γ-motoneurons. Alternatively, it has been suggested that a reduction in neurotransmitter release at the Ia afferent terminal ending [51] or an increase in the discharge of group IV joint afferents [45] may contribute to γ-loop dysfunction [14]. Future studies may wish to examine these and other mechanisms in more detail. If γ-loop dysfunction is simply caused by a loss of excitatory input from joint afferents to quadriceps γ-motoneurons, then the afferent portion of the pathway should be unaffected. If this is the case, short-duration vibration applied during a strong voluntary contraction may be able to artificially restore transmission in Ia afferents, enhancing quadriceps muscle activation [28]. A study testing this hypothesis is currently being undertaken in our laboratory. In addition to the results presented in the current study, quadriceps γ-loop dysfunction has been observed after ACL injury [32,35], after ACL reconstructive surgery [36,42] and in elderly patients hospitalised after a fall [52]. Importantly, the mechanisms explaining γ-loop dysfunction may be different in different populations. Obtaining a better understanding of its underlying causes could have important implications in the rehabilitation of these patients.

The article "Mechanisms of quadriceps muscle weakness in knee joint osteoarthritis: the effects of prolonged vibration on torque and muscle activation in osteoarthritic and healthy control subjects" was published in 2011. Journal: Arthritis Res Ther.

In the current study, quadriceps strength was reduced by 32% in the OA group compared with an age-matched and gender-matched control group. This compares well with previous studies in the literature that have observed quadriceps strength deficits of 20 to 45% in people with knee joint OA [1-3]. Part of this weakness is due to muscle atrophy and part due to AMI. At least in individuals with severe OA, AMI appears to account for a greater portion of quadriceps weakness than muscle atrophy [13]. Comparative data does not exist for individuals in earlier stages of the disease. However, Pap and colleagues found the magnitude of quadriceps AMI to be slightly higher in OA patients with moderate joint degeneration compared with those with more severe and widespread joint damage [53]. Furthermore, one should consider that an inability to fully activate the muscle is likely to contribute to a portion of the atrophy anyway [15,19]. Thus, AMI may have direct and indirect effects on quadriceps muscle weakness.

While prolonged vibration is a useful neurophysiological tool to explore the function of the γ-loop, it does not allow us to accurately determine the contribution of γ-loop dysfunction to the overall magnitude of AMI, or quadriceps weakness. AMI can be severe in individuals with knee OA, with quadriceps voluntary activation deficits of 25 to 35% observed [2,46,54]. Although the ~8% reduction in post-vibration quadriceps torque seen in the control group may suggest that the γ-loop makes a relatively small contribution to the overall level of AMI, this is not necessarily true.

Microneurography studies have demonstrated that the firing rate of most Ia afferent fibres is depressed following vibration, and the spindle response to stretch is reduced by ~25% [55]. Furthermore, Hoffman reflex amplitude - which is partly determined by Ia afferent transmission - is reduced by ~30 to 40% following prolonged vibration [56]. However, we cannot be sure what portion of the Ia afferent drive is impaired in pathological populations with γ-loop dysfunction. We can simply observe that prolonged vibration has no additional effect on OA subjects' ability to activate their quadriceps, which suggests these individuals have a pre-existing impairment in Ia afferent drive of at least the same level as that produced by 20 minutes of vibration. For example, it may be that ~30% of the effective Ia afferent drive is impaired by prolonged vibration but that in OA subjects with γ-loop dysfunction ~80% of the effective Ia afferent drive is impaired. In this case, prolonged vibration may have no additional effect on quadriceps activation in OA subjects but neither would the change in quadriceps activation observed in healthy controls represent the true effect of γ-loop dysfunction on quadriceps activation in a pathological population (which would be greater).

The article "Mechanisms of quadriceps muscle weakness in knee joint osteoarthritis: the effects of prolonged vibration on torque and muscle activation in osteoarthritic and healthy control subjects" was published in 2011. Journal: Arthritis Res Ther.

Furthermore, because AMI is caused by activity in multiple inhibitory pathways [14] the influence of γ-loop dysfunction may be underestimated in individuals with OA. This is due to spatial facilitation and the all-or-nothing nature of α-motoneuron depolarisation. While firing of a discrete number of α-motoneurons may be completely prevented by a given inhibitory input, others will only be partially inhibited and are still able to depolarise [57]. However, when two (or more) forms of inhibitory/disfacilitatory input are present, the partial inhibition produced by each input is often sufficient to prevent depolarisation of a greater number of α-motoneurons, so that the total inhibition is greater than the algebraic sum of the individual inhibitory/disfacilitatory inputs [58]. In this way, even if prolonged vibration exactly mimicked the loss of Ia afferent drive produced by γ-loop dysfunction, the effects of γ-loop dysfunction on quadriceps activation may be far greater in a pathological population than the effects of prolonged vibration on quadriceps activation in healthy controls.

A limitation of the current study is that we did not confirm the presence of a quadriceps activation deficit in the OA group using techniques such as burst superimposition or interpolated twitch. As such, it could be argued that, despite evidence of γ-loop dysfunction, the OA subjects in the present study may have learnt to fully activate their quadriceps in the absence of full excitatory input from Ia afferents. While this is theoretically possible, we consider it unlikely. The majority of studies that have assessed quadriceps activation in people with knee joint OA have found clear evidence of AMI [59]. Those studies where quadriceps activation deficits are equivocal all used burst superimposition to calculate quadriceps central activation ratios [41,60-64]. The central activation ratio has consistently been shown to overestimate quadriceps activation compared with interpolated twitch [65-68], while even interpolated twitch has been suggested to overestimate true muscle activation [69] (thus underestimating AMI).

## Conclusions

The results of the present study suggest that γ-loop dysfunction contributes to quadriceps AMI in individuals with knee joint OA. The subsequent loss of Ia afferent feedback during strong voluntary contractions may partially explain the marked quadriceps weakness and atrophy that is often observed in this population. Quadriceps weakness is clinically important in individuals with OA because it associated with physical disability [2-5], an increased rate of loading at the knee [7,8] and has been identified as a risk factor for the initiation and progression of joint degeneration [9-11]. Future research should aim to gain a better understanding of the mechanisms underlying γ-loop dysfunction and explore how these may differ across pathologies.

The article "Mechanisms of quadriceps muscle weakness in knee joint osteoarthritis: the effects of prolonged vibration on torque and muscle activation in osteoarthritic and healthy control subjects" was published in 2011. Journal: Arthritis Res Ther.

## Abbreviations

ACL: anterior cruciate ligament; AMI: arthrogenic muscle inhibition; EMG: electromyography; MVC: maximum-effort voluntary contraction; Nm: Newton metres; OA: osteoarthritis; RMS: root mean square.

## Competing interests

The authors declare that they have no competing interests.

## Authors' contributions

DAR was involved in the conception and design of the study, the collection, analysis and interpretation of the data, and the drafting and revision of the manuscript. PJM was involved in the conception and design of the study, the analysis and interpretation of the data, and the revision of the manuscript. GNL was involved in the conception and design of the study, the collection and interpretation of the data, and the revision of the manuscript. All the authors read and approved this manuscript for publication.
